# Medical Image Fusion Based on Low-Level Features

**DOI:** 10.1155/2021/8798003

**Published:** 2021-06-10

**Authors:** Yongxin Zhang, Chenrui Guo, Peng Zhao

**Affiliations:** College of Information Technology, Luoyang Normal University, Luoyang 471934, China

## Abstract

Medical image fusion is an important technique to address the limited depth of the optical lens for a completely informative focused image. It can well improve the accuracy of diagnosis and assessment of medical problems. However, the difficulty of many traditional fusion methods in preserving all the significant features of the source images compromises the clinical accuracy of medical problems. Thus, we propose a novel medical image fusion method with a low-level feature to deal with the problem. We decompose the source images into base layers and detail layers with local binary pattern operators for obtaining low-level features. The low-level features of the base and detail layers are applied to construct weight maps by using saliency detection. The weight map optimized by fast guided filtering guides the fusion of base and detail layers to maintain the spatial consistency between the source images and their corresponding layers. The recombination of the fused base and detail layers constructs the final fused image. The experimental results demonstrated that the proposed method achieved a state-of-the-art performance for multifocus images.

## 1. Introduction

The depth-of-field limitations may potentially limit the complete and accurate understanding of the medical problem of the human body, organs, and cells and even the performance of medical diagnostics and analysis [1–3]. Medical image fusion is an essential technique for combining multiple images with complementary information to provide more comprehensive descriptions of the medical problems [4]. To date, medical image fusion has become a relevant research field due to its efficiency and wide applications in medical analysis. The growing appeal of high-performance medical diagnostic devices prompts the development of low-cost computing and imaging techniques. There are many medical image fusion methods proposed to address the problems mentioned above. These methods include two categories: spatial domain methods and transform domain methods [5].

The spatial domain methods deal with pixels or regions in spatial domains directly based on the pixel intensities [6]. The fundamental problem of spatial domain methods is the selection of the clearest image pixels or regions from the source images in order to construct the fused image. The regions with greater energy or larger changes of pixels are considered to be in focus during the fusion process. The spatial domain methods mainly include pixel-based methods [6–8] and region-based methods [9–11]. These methods are simple and fast. However, the pixel-based methods are sensitive to noise, which may potentially lead to the incorrect choice of pixels. Due to difficulties in the selections of block sizes or segmentation algorithms [12, 13], the region-based methods suffer from blocking artifacts. Also, the visual quality of the final fused image could be compromised when blur and sharp pixels are segmented to the focused regions [5].

The transform domain methods deal with the coefficients of the transformed source images in the transform domain. The transform domain methods that approximate and detail coefficients at different scales integrate these coefficients to new multiscale representation by employing various fusion rules. And finally, an inverse transformation is performed on these coefficients to reconstruct a fused image [4]. Based on the hypothesis that the greater the frequency content in the transform domain, the higher the corresponding contrasts in the spatial domain, the regions with greater coefficients of high frequency are accepted as being in focus during the fusion process. These methods mainly include the following: the Laplacian pyramid (LAP) [14], discrete wavelet transform (DWT) [15], curvelet transform (CVT) [16], contourlet transform (CT) [17], and non-subsampled contourlet (NSCT) [18]. These methods can achieve better signal-to-noise ratios [19]. However, they suffer from time and space consumption, loss of contrast, selection of the decomposition level, and decomposition type. The simple fusion rules of these methods cannot always successfully identify the detailed and structured information from coefficients, and may cause the degradation of image quality [20]. Due to spatial inconsistencies, these methods are unable to effectively preserve the edge and texture information, which may lead to halo artifacts near the edges, as well as spurious data and distortions.

In recent years, deep learning as a novel technique is applied to medical image fusion for better fusion performance. Liu et al. [21] fused the medical image by integrating MCA and convolutional sparse representation (CSR) into a unified optimization framework. It can outperform some benchmarking and state-of-the-art SR-based fusion methods. Xia et al. [22] proposed a novel fusion scheme for multimodal medical images which utilizes both the features of the multiscale transformation and deep convolutional neural network. Hou et al. [23] designs a novel fusion scheme for CT and MRI medical images based on convolutional neural networks and a dual-channel spiking cortical model. Ding et al. [24] fused medical images by combining convolutional neural networks and non-subsampled shear-let transform to simultaneously cover the advantages of them both for medical image fusion. Wang et al. [25] proposed a medical image algorithm based on the Siamese convolutional network and contrast pyramid. These algorithms can effectively preserve the detailed structure information of source images and achieve good human visual effects. These methods have achieved better fusion performance. However, the need for tuning millions of parameters during the training stage, as well as the difficulty of exploration, seriously affected the fusion quality.

Recently, edge-preserving filter-based fusion methods are introduced to solve the problems mentioned above and they simplify the representation of source images while retaining the robust edges [26]. They include the guided filtering method [27], *L*_0_ gradient minimization method [28], cross-bilateral filter (BF) method [29], weighted least square filter method [30], and rolling guidance method [31]. The guided filtering method retained the spatial consistency of the base and detail layers by using a weighted average technique. The *L*_0_ gradient minimization method preserved and enhanced human visual system interests by using visual weight maps. The cross-bilateral filter method fused the source images by using the detailed information of the source images. The rolling guidance method prevented noise and image distortion through the spiking cortical model, while the iterative guided filtering method suppressed the noise by using a guided filter in an iterative mode. All these methods achieved excellent performance for medical image fusion. This paper mainly focuses on the improvement of the conventional image fusion method.

As we know, low-level features such as color, texture, edge shape, and structure are the significant features for image representation. These features are the key to image saliency detection and image understanding. It is significant for medical analysis and decisions according to medical images. The low-level feature is the salient feature for focused region detection. It can improve the accuracy of the focused region detection by using low-level features. Then, more structured and detailed information can be transferred into the fused image from the source images. Thus, high-quality fusion result can be obtained. To further improve the medical image fusion quality by using a low-level feature, we propose a novel medical image fusion scheme with a low-level feature. In the beginning, the proposed method decomposes the source images into base and detail layers by using local binary patterns operators for the low-level feature. Then, weight maps of the base and detail layers are constructed based on the low-level feature. Thirdly, the base and detail layers are fused according to the optimized weight map with a fast guided filter. Finally, the fused base and detail layers are combined to produce the final fused image. The fast guided filter (FGF) is one of several popular filters for edge-preserving smoothing, which is independent of the filter size. Due to its flexibility and speed of computation, it is feasible to use in different real-time applications. The objective of this paper is to investigate its potential applications in medical image fusion.

This paper's main contributions fell into the following three points:

1. We propose a novel multifocus image fusion method with a low-level feature
2. We propose a novel weight construction method according to low-level feature saliency and spatial context
3. We extract the low-level feature by using local binary patterns operators

The rest of this paper is organized as follows: Section 2 explains the basic concept of FGF which discusses its feasibility and advantages for medical image fusion, whereas Section 3 defines the fusion method with FGF.  Section 4 discusses experimental results followed by conclusions and future work in Section 5.

## 2. Related Works

### 2.1. Fast Guided Filter

FGF is one of several popular techniques for edge-aware image filtering, whose computing time is independent of the filter size [26]. In this study, the FGF is applied to medical image fusion. In theory, FGF is driven by a local linear model and the relation between the guidance image *I* and filter output image *O* in a local square window *ω*_*k*_ centered at the pixel *k* is defined as follows:

(1) $$\begin{array}{c} O_{i}=a_{k}I_{i}+b_{k},\;\forall i\in \omega_{k}, \end{array}$$

where *i* denotes a pixel and *a*_*k*_ and *b*_*k*_ are liner coefficients in *ω*_*k*_. The size of *ω*_*k*_ is (2*r* + 1)(2*r* + 1). The linear coefficients *a*_*k*_ and *b*_*k*_ are used to minimize the squared difference between the filter input image *P* and the filter output image *O*. The linear coefficients *a*_*k*_ and *b*_*k*_ can be obtained by linear regression as follows:

(2) $$\begin{array}{c} a_{k}=\frac{\left(1/\left|\omega \right|\right)\sum_{i\in \omega_{k}}I_{i}P_{i}-u_{k}{\bar{P}}_{k}}{\sigma_{k}^{2}+\varepsilon },\\ b_{k}={\bar{P}}_{k}-a_{k}b_{k}, \end{array}$$

where *u*_*k*_ and *σ*_*k*_ are the mean and variance of *I* in the window *ω*_*k*_, respectively, |*ω*| denotes the pixel number in *k*, and $\bar{P}$ denotes the mean value of *P* in *ω*_*k*_. *ε* is a regularization parameter, which controls the degree of smoothness on *P*. The filtering output image *O* is defined as follows:

(3) $$\begin{array}{c} O_{i}={\bar{a}}_{i}I_{i}+{\bar{b}}_{i}, \end{array}$$

where ${\bar{a}}_{i}$ and ${\bar{b}}_{i}$ are two smoothed maps and denote the mean value of *a* and *b*, respectively, in *ω*_*i*_. The main computation of FGF is for the smoothed maps of ${\bar{a}}_{i}$ and ${\bar{b}}_{i}$. In order to improve the computational efficiency, all the box filters are performed on the low-resolution maps. Moreover, ${\bar{a}}_{i}$ and ${\bar{b}}_{i}$ are bilinearly upsampled to the original size.

### 2.2. Feasible and Superiority

Figure 1 lists the comparison of BF and FGF for image filtering. The enlarged region of the filtering results for the source image demonstrates that FGF can well inhabit gradient-reversal artifacts and preserve the low-level features.

It is known that a suitable fusion method should transfer most of the useful low-level feature, such as edges, texture, and structure information, from the source images to the fused image. FGF is a novel edge-preserving smoothing technique, which can effectively remove noise, weak edges, and small details while preserving the overall low-level features of an image. Activity level measurements and focus regions or pixel extractions are two essential problems affecting the fusion quality. As mentioned above, the transform domain-based fusion methods use predesigned bases to represent the source images. The spatial domain-based fusion methods use activity-level measurements based on high-pass spatial filtering. FGF is able to well preserve the low-level feature such as colors, boundary, structures, edges, and textures corresponding to those of the source images. The low-level feature of base and detail layers can be used to perform more effective activity-level measurements and accurately discriminate the focused regions from the defocused regions. The fusion of the source images can be transformed into the subfusion of base and detail layers. FGF can well extract the low-level feature from the source images. Therefore, it was determined that it is feasible to apply FGF to medical image fusion. The advantages of the FGF-based fusion method over other existing methods are fourfold: (1) FGF can effectively suppress gradient-reversal artifacts [15] and produce visually pleasing edge profiles, (2) FGF is independent of the filter size and well suited for real applications with highly computed efficiency, (3) FGF is flexible and easy to implement, and (4) the FGF-based fusion method can be adapted to different field applications.

Considering the advantages of FGF mentioned above, we propose a novel FGF-based fusion method to extract the low-level features for saliency map construction and guide the medical image fusion, as detailed in Section 3.

## 3. Proposed Approach

### 3.1. Fusion Algorithm

We assumed that there are two registered source images *I*_1_ and *I*_2_, which are preregistered. As shown in Figure 2, the proposed fusion algorithm consists of four main steps:

**Step 1 .**

(two-scale image decomposition).

The local binary pattern (LBP) operators [32] are applied to decompose the source images *I*_1_,*I*_2_ into base layers *B*_1_,*B*_2_ and detail layers *D*_1_,*D*_2_ respectively. It can be defined as follows:

(4) $$\begin{array}{c} I=B+D, \end{array}$$

where *I* is the source image, *B* is the base layer of *I*, and *D* is the detail layer of *I*.

**Step 2 .**

(construction of decision map for subfusion).

Laplacian filtering (LF) and Gaussian low-pass filtering (GLF) are performed on the source images *I*_1_, *I*_2_ to obtain the saliency maps *S*_1_ and *S*_2_, respectively, which are compared to construct weight maps *P*_1_ and *P*_2_, respectively. Weight maps *P*_1_ and *P*_2_ are optimized for *W*_1_^*B*^, *W*_2_^*B*^ and *W*_1_^*D*^, *W*_2_^*D*^, respectively, with FGF guided by source images *I*_1_ and *I*_2_, respectively.

**Step 3 .**

(subfusion of different layers).

Following the fusion rules and optimized weight maps, *B*_1_ and *B*_2_ are integrated to obtain *F*_*B*_, which denotes the fused base layer*D*_1_. Moreover, *D*_2_ is integrated to obtain the fused detail layer *F*_*D*_.

**Step 4 .**

(two-scale image reconstruction).

*F*_*B*_ and *F*_*D*_ are combined to construct the final fused image *F*.

(5) $$\begin{array}{c} F=F_{B}+F_{D}. \end{array}$$

### 3.2. Fusion Rule

As mentioned above, the low-level features of the source images such as colors, boundary, structures, edges, and textures can be used to perform more effective activity-level measurements and accurately discriminate the focused regions from the defocused regions. The relationship between the source images “skull” and their corresponding layers is shown in Figure 3. It can be seen that the low-level features of the source images are corresponding to the low-level feature of different layers, such as the structure, the textures, and the edges of the tissue.

In order to measure the activity level, we apply Laplacian filtering and Gaussian low-pass filtering to detect the salient feature and construct the saliency maps of the source images. The Laplacian filter highlights the change in light intensity surrounding a pixel. It can extract the outline of the target and generalize the details. Laplacian filtering is used for obtaining the high-pass component of the source image. Gaussian low-pass filter is a linear smoothing filter, which is suitable for eliminating Gaussian noise and is widely used in the denoising process of image processing. Gaussian filtering is a process of weighted averaging of the entire image. The value of each pixel is obtained by weighted averaging of itself and other pixel values in the neighborhood. In this study, Gaussian low-pass filtering is used for computing the local average of the absolute value of the obtained high-pass component, which constructs the saliency maps *S*. The saliency map is defined as follows:

(6) $$\begin{array}{c} S=I*L*G, \end{array}$$

where *S* is the saliency map. *L* is the Laplacian filtering. *G* is Gaussian low-pass filtering. The obtained saliency maps represent the saliency level of detail information. The pixel maximum of the saliency maps is computed to construct the corresponding weight maps *P*, which are defined as follows:

(7) $$\begin{array}{c} P_{1}\left(i,j\right)=\left\{\begin{array}{c} 1,\;S_{1}\left(i,j\right)\geq S_{2}\left(i,j\right),\\ 0,\;\text{otherwise}, \end{array}\right.\\ P_{2}\left(i,j\right)=\left\{\begin{array}{c} 1,\;S_{2}\left(i,j\right)\geq S_{1}\left(i,j\right),\\ 0,\;\text{otherwise}, \end{array}\right. \end{array}$$

where “1” in weight maps indicated that the pixel location (*i*, *j*) in source images was in focus. However, the weight maps are not well consistent with the object boundaries in the source images. It may produce artifacts in the fused image. As shown in Figure 3, the base layers are spatially smooth and the detail layers have large moment of detailed information. Spatial consistency demands that those pixels with similar color or brightness tend to have similar weights. Thus, the weights for base layers should be spatially smooth and the weights for detail layers should be sharp. FGF is applied to optimize the binary maps with the source image *I* serving as a guidance image. A large filter size and large blur degree are used for the fusion of base layers. A small filter size and small blur degree are used for the fusion of detail layers. Optimized weight maps *W* are defined as follows:

(8) $$\begin{array}{c} W=FGF\left(P,I\right). \end{array}$$

Then, the base and detail layers obtained by using LBP are fused with optimized weighted maps *W*. The multilayers of the source images are fused as follows:

(9) $$\begin{array}{c} F_{B}=W_{1}^{B}B_{1}+W_{2}^{B}B_{2},\\ F_{D}=W_{1}^{D}D_{1}+W_{2}^{D}D_{2}, \end{array}$$

where *F*_*B*_ and *F*_*D*_ represent the fused base layer and the fused detail layer, respectively.

## 4. Experimental Results

In this section, some commonly used testing image sets are used to assess the performance of the proposed method. To be more objective in the performance assessment, the proposed method is compared with some of the existing fusion algorithms in terms of visual quality and quantitative evaluation.

### 4.1. Experimental Settings

#### 4.1.1. Testing Images

In the experiments, nine pairs of medical images of the database [21, 33] are used as the testing image sets, as shown in Figure 4. These images have a resolution of 256 × 256 pixels and 256 levels, except for the ninth group of images that have a resolution of 464 × 464.

#### 4.1.2. Compared Algorithms

These comparison methods include traditional fusion methods, as well as recently proposed fusion methods. The traditional fusion methods are the Laplacian pyramid- (LAP-) based fusion algorithm, discrete wavelet transform- (DWT-) based fusion algorithm, and non-subsampled contourlet- (NSCT-) based fusion algorithm. The recently proposed fusion methods included cartoon-texture decomposition- (CTD-) based fusion algorithm [34], multiscale image decomposition- (MSID-) based fusion algorithm [35], cross-bilateral filtering- (CBF-) based fusion algorithm [24], and guided filtering fusion- (GFF-) based algorithm [22]. The compared algorithms and proposed algorithm are all programmed in MATLAB language, and all the experiments are conducted with MATLAB R2011b in a Windows environment, on a computer with an Intel Core (TM) i7-4770 and 4G memory. Due to the lack of a source code, this study uses the Eduardo Fernandez Canga's MATLAB image fusion toolbox [36] as the reference for the LAP and DWT. The NSCT toolbox [37] is used as a reference for the NSCT. The toolboxes of CTD and FGF available from [21, 34] are used for the CTD and the proposed fusion methods. The source codes of the GFF are derived from [38] as the reference for the fusion based on the GFF. The evaluation toolboxes are taken from [39] and used for the fusion performance evaluations.

#### 4.1.3. Parameter Setting

The decomposition level of the DWT was 4. Also, the pyramid filter “9–7” and orientation filter “7–9” with {4, 4, 3} levels of decomposition were set for the NSCT. The parameters of the recently proposed fusion methods, such as CTD, MSID, CBF, and GFF, are found to be the same with the corresponding papers. The local window radius and the regularization parameters of the FGF are set as *r*_1_ = 45, *r*_2_ = 7.5, *ε*_1_ = 0.25, and *ε*_2_ = 10^‐6^.

#### 4.1.4. Evaluation Metrics

Four commonly used evaluation metrics, i.e., mean square error (MSE), mutual information (MI) [40], *Q*^*AB*/*F*^ [41], and *Q*_*Y*_ [42], are used to evaluate the effectiveness of the proposed method. These metrics measure the information preservation ability of the fusion method. MSE measures the similarity between the source images and the fused image. MI measures the degree of the information transferred from source images to the fused image. *Q*^*AB*/*F*^ measures the amount of edge information transferred from the source images to the fused image. *Q*_*Y*_ measures the amount of the structural information preserved from the source images to the fused image by using structural similarity. The larger value of these metrics (MI, *Q*_*Y*_, and *Q*^*AB*/*F*^) and the lower value of MSE represent a large amount of information preserved from the source images and signifies a better fusion performance.

### 4.2. Quality Assessment

For assessing the visual quality of fusion results obtained by different methods, Figures 5 and 6 show the fusion results of “MI-1” and their corresponding enlarge regions. Figures 7 and 8 show the fusion results of “MI-4” and their corresponding enlarged regions. Figures 9 and 10 show the fusion results of “MI-5” and their corresponding enlarged regions. Figures 11 and 12 show the fusion results of “MI-8” and their corresponding enlarged regions.

LAP can well extract low-level features from the source images except for suffering from the instability of the relationship of decomposition coefficients between different levels. The extraction of point-wise singularities for DWT is better than that of in-line singularities. The shift invariance of NSCT improves the extraction capacity of low-level features from the source images. However, a large number of decomposition coefficients consume more memory space and processing time. Moreover, LAP, DWT, and NSCT produce the fusion results in the transform domain by processing the transform coefficients. However, the spatial inconsistency compromises fusion performance. The fusion results demonstrate noticeable blurs, such as the edge of the soft tissue of the brain (Figures 5(a)–5(c)), the edge of the skull (Figures 7(a)–7(c), 9(a)–9(c), and 11(a)–11(c)), the upper edge of the enlarged detail regions (Figures 6(a)–6(c), 8(a)–8(c), 10(a)–10(c), and 12(a)–12(c)).

CTD is an improved technique for the problems of L1-regularized optimization. It can well extract the low-level features such as structural patterns and latent detail information of source images with cartoon-texture decomposition. The source image can be split into cartoon components and texture components with a split Bregman algorithm. The salient low-level features are compared to construct the decision map for the fusion of cartoon and texture components. However, the construction of the decision map for cartoon and texture components is affected by the imprecise morphological operation, such as erosion and dilation. Thus, the low-level feature of the source image cannot be well transferred to the fused image. The corresponding artifacts of CTD can be seen in the edge regions of the enlarged detail regions (Figures 6(a)–6(d)).

MSID is based on saliency detection and multiscale image decomposition. MSID is efficient to emphasize visual saliency by extracting low-level features. It can improve the capacity of focused region detection. Weight maps of this algorithm are capable of detecting and identifying focused and defocused regions of the source images. However, the weight maps for final approximation layer compromise the fusion performance and produce the noticeable blurs such as the blurred edge of the soft tissue of the brain (Figure 5(e)), the apparent blur edge of the skull (Figures 7(e), 9(e), and 11(e)), the incomplete edge, and low contrast in the enlarged detail regions (Figures 6(e), 8(e), 10(e), and 12(e)).

The cross-bilateral filter considers both gray-level similarities and geometric closeness of the neighboring pixels without smoothing edges, but it uses one image for finding the kernel and the other to the filter and vice versa. CBF applies joint bilateral filtering to extract low-level features for suppressing the gradient reversal artifacts of the bilateral filter. It fuses source images by weighted average using the weights computed from the detail layers. However, the fusion of different layers based on weight maps may be affected by the combination of the pixels with different intensities. The low contrast and visible blurs can be seen in the fused images, such as the incompleteness of the soft tissue of the brain (Figure 5(f)), the obvious blur edge of the skull (Figures 7(f), 9(f), and 11(f)), and the low contrast in the enlarged detail regions (Figures 6(f), 8(f), 10(e), and 12(f)).

GFF is based on a two-scale decomposition of an image into a base layer containing large-scale variations in intensity and a detail layer capturing small-scale details. GFF is an efficient fusion method. It combines pixel saliency and the spatial context for medical image fusion. It improves the fusion performance by combining the different layers with optimized saliency maps constructed from the low-level features. However, the weight map operations used in the fusion process can result in the loss of some low-level features of the source images due to inaccurate weight values. It can be seen in the fused images, such as the blurring artifacts, e.g., the corresponding enlarged detail regions (Figures 8(g) and 12(g)).

The proposed method decomposes the source images into base layers and detail layers by using local binary pattern operators. The saliency low-level features such as texture, edge, and structure are extracted by Laplacian filtering and Gaussian low-pass filtering. These features are compared to construct the saliency maps, which optimized to weight maps for the fusion of different layers by using fast guided filtering. Fast guided filtering is adopted as a local filtering for optimization of the weight maps. Different filter sizes and blur degrees control the pixel saliency and spatial consistency by adjusting the value of the parameters in the fast guided filter. Different layers are fused with corresponding weight maps based on the guidance of the source images. The pixel saliency and spatial consistency can be well improved, which ensures the better fusion performance of the proposed method. The visual quality assessment of the fusion results obtained by different methods has demonstrated that the proposed method has achieved better visual quality than that of other methods. The detailed visual information of the fusion results demonstrates the superiority of the proposed method.

### 4.3. Quantitative Analysis

In order to compare the fusion performance of different fusion methods, four evaluated metrics mentioned above are applied to the fused medical images. These metric values are listed in Table 1. The bar charts of the average values of the three metrics (MI, *Q*_*Y*_, and *Q*^*AB*/*F*^) in Table 1 are shown in Figure 13. The average running time of the compared algorithms is listed in Table 2.

It is easy to see that the MI and *Q*^*AB*/*F*^ values of CTD and the proposed are higher than those of other fusion methods. The *Q*^*AB*/*F*^ values of LAP and DWT are higher than those of NSCT. The *Q*^*AB*/*F*^ values of NSCT are lower than those of other fusion methods. The *Q*_*Y*_ and MI values of MSID are lower than those of other fusion methods. The MSE values of NSCT are higher than those of other fusion methods. The MSE values of the proposed method are lower than those of other fusion methods. The values of Table 1 and the change of the trend chart (MI, *Q*_*Y*_, and *Q*^*AB*/*F*^) demonstrate the proposed method has achieved better performance. Table 2 demonstrates that the NSCT required the longest computational times, followed by CBF and CTD. The reason is that the processing of coefficients consumes most of the fusion time. The statistic model of CBF consumes most of the fusion time. The sliding window of CTD consumes the running time. As previously mentioned, this study demonstrates that the proposed method costs little time for the medical images.

## 5. Conclusion

This study presented a novel medical image fusion method based on the low-level feature. The fast guided filtering is applied to the saliency map of the source images to construct the weight map of the multilayers of the source images. The base and detail layers obtained by local binary pattern operators are fused according to their corresponding weight maps, and the fused base and detail layers are combined to produce the final fused image. This study's experiments are performed on nine pairs of medical images. The experimental results demonstrate that the proposed method obtains a state-of-the-art performance in both qualitative and quantitative evaluations. The optimization in parameter adaptability is exciting and worthwhile for further investigations.

## Figures and Tables

**Figure 1:** Comparison of different filters.

**Figure 2:** Algorithm framework.

**Figure 3:** Relationship between the source images and their corresponding layers.

**Figure 4:** Test images used in the experiments.

**Figure 5:** Experimental results Aof “MI-1” obtained using different fusion methods.

**Figure 6:** Enlarged regions from fusion results of “MI-1” obtained using different fusion methods.

**Figure 7:** Experimental results of “MI-4” obtained using different fusion methods.

**Figure 8:** Enlarged regions from fusion results of “MI-4” obtained using different fusion methods.

**Figure 9:** Experimental results of “MI-5” obtained using different fusion methods.

**Figure 10:** Enlarged regions from fusion results of “MI-5” obtained using different fusion methods.

**Figure 11:** Experimental results of “MI-8” obtained using different fusion methods.

**Figure 12:** Enlarged regions from fusion results of “MI-8” obtained using different fusion methods.

**Figure 13:** Average metric values of different methods for medical images.

**(a):** 

Method	MI-1				MI-2				MI-3			
	MI	*Q*_*Y*_	*Q* ^*AB*/*F*^	MSE	MI	*Q*_*Y*_	*Q* ^*AB*/*F*^	MSE	MI	*Q*_*Y*_	*Q* ^*AB*/*F*^	MSE
LAP	2.178	0.675	0.727	57.741	2.068	0.872	0.739	45.730	2.609	0.903	0.627	44.14481354
DWT	2.931	0.827	0.611	79.965	3.129	0.961	0.787	54.263	2.599	0.832	0.565	53.49580383
NSCT	2.177	0.620	0.465	90.939	2.825	0.584	0.793	65.552	2.796	0.566	0.612	65.61071777
CTD	5.914	0.943	0.664	74.500	3.940	0.936	0.830	51.555	4.483	0.975	0.673	41.62849426
MSID	2.195	0.616	0.499	59.269	1.582	0.844	0.496	43.559	2.232	0.848	0.436	44.26103973
CBF	4.412	0.924	0.775	74.774	2.837	0.928	0.776	51.407	2.904	0.905	0.626	42.7221756
GFF	3.259	0.887	0.780	78.395	2.157	0.768	0.797	49.230	2.669	0.751	0.639	42.53501129
Proposed	**6.032**	**0.959**	**0.820**	**46.075**	**4.063**	**0.964**	**0.851**	**43.405**	**4.574**	**0.988**	**0.737**	**38.040**77911

**(b):** 

	MI-4				MI-5				MI-6			
LAP	2.739	0.901	0.607	50.271	2.414	0.897	0.656	40.721	2.671	0.897	0.614	46.824
DWT	2.690	0.834	0.535	55.560	2.541	0.850	0.614	51.070	2.670	0.829	0.551	55.585
NSCT	2.824	0.540	0.577	70.298	2.684	0.543	0.667	62.506	2.793	0.558	0.573	69.043
CTD	4.779	0.959	0.665	30.326	4.101	0.921	0.695	41.111	4.673	0.967	0.649	44.490
MSID	2.431	0.850	0.434	45.375	2.093	0.858	0.465	40.912	2.293	0.845	0.430	45.553
CBF	2.945	0.892	0.594	43.758	2.765	0.909	0.656	40.511	2.928	0.890	0.606	44.624
GFF	2.762	0.756	0.625	41.943	2.462	0.741	0.654	39.297	2.642	0.742	0.617	44.171
Proposed	**4.863**	**0.974**	**0.692**	**36.298**	**4.113**	**0.994**	**0.736**	**38.885**	**4.694**	**0.988**	**0.712**	**43.713**

**(c):** 

	MI-7				MI-8				MI-9			
LAP	2.803	0.900	0.613	46.924	2.888	0.907	0.624	42.013	3.249	0.796	0.614	33.56437
DWT	2.783	0.817	0.558	51.125	2.732	0.799	0.553	49.897	3.197	0.794	0.490	51.27275
NSCT	2.976	0.577	0.624	66.102	2.987	0.584	0.630	63.085	3.318	0.779	0.529	55.56722
CTD	4.887	0.982	0.677	39.625	4.848	0.979	0.683	37.383	3.704	0.870	0.593	47.99319
MSID	2.514	0.848	0.437	43.682	2.575	0.851	0.460	40.935	3.112	0.725	0.445	34.95961
CBF	3.043	0.891	0.597	41.760	3.075	0.897	0.613	38.117	4.378	0.880	0.616	26.81659
GFF	2.786	0.755	0.623	41.034	2.849	0.755	0.634	38.010	4.061	0.910	0.675	27.27437
Proposed	**4.926**	**0.998**	**0.720**	**37.291**	**4.927**	**0.994**	**0.711**	**34.563**	**4.112**	**0.983**	**0.703**	**25.441**2

**Table 2:** Average running time of different fusion methods for medical images.

Method	LAP	DWT	NSCT	CTD	MSID	CBF	GFF	Proposed
Time (s)	0.254	0.105	20.750	3.140	1.484	11.746	0.162	**0.142**

## Data Availability

The medical image data used to support the findings of this study have been deposited in references [20, 30].
